The article "Measuring the Effect of Smoking or Tobacco Use on Vertigo Among the Adult Population in the Kingdom of Saudi Arabia" was retracted in 2023. Reasons: errors in the methods; unreliable results or conclusions; concerns about the results or conclusions.

# Measuring the Effect of Smoking or Tobacco Use on Vertigo Among the Adult Population in the Kingdom of Saudi Arabia

**DOI:** 10.7759/cureus.38516

**Published:** 2023-05-03

**Authors:** Mohahmmed Alateeq, Tamara A Hafiz, Osama Alnizari

**Affiliations:** 1 Otolaryngology-Head and Neck Surgery, University of Hail College of Medicine, Hail, SAU; 2 Public Health, Umm Al-Qura University, Makkah, SAU; 3 Family Medicine, University of Hail College of Medicine, Hail, SAU

**Keywords:** tobacco, saudi arabia, tinnitus, hearing impairment, smoking

## Abstract

Background

Smoking is widespread at all ages in Saudi society. In addition, complaints of vertigo are common. A key problem is how smoking affects vertigo and, thus, quality of life. Researchers have investigated the association between smoking and vertigo and found that smoking may be a risk factor for vertigo, but this association is not clear. The current study aims to investigate the association between smoking and vertigo.

Materials and methods

We conducted a cross-sectional study from March 2022 to January 2023 to investigate the effect of smoking on vertigo in Saudi Arabia’s adult population.

Results

We found that smokers were more prone to vertigo than non-smokers. In addition, the severity of vertigo increases as the number of cigarettes smoked or the length of time in years that the person has smoked increases.

Conclusion

The findings of the study should inspire more research into the impact of demographic factors on vertigo among smokers.

## Introduction

Smoking tobacco poses a major risk to health [1] and ranks among the top avoidable causes of death worldwide [2]. According to studies, tobacco use increases the risk of six out of the top eight global killers [3]. Similar studies have revealed that tobacco use results in the deaths of about eight million individuals annually [4]. In addition, smoking tobacco can cause a number of illnesses, including cancer. The most common cancer is lung cancer, which is the primary cause of death in the United States [5], as well as cardiovascular disease [6] and cerebrovascular disease [7].

Because vertigo is a possible symptom of any of these conditions, it is plausible to assume that smoking is related to vertigo. Additionally, it is unknown if smoking poses a separate risk for vertigo. Researchers in Saudi Arabia found that the country has a smoking prevalence between 2.4% and 52.3% [8]. Smoking rates range from 12.8% to 29.8% among schoolchildren, from 2.4% to 37% among college students, and from 11.6% to 52.3% among adults. Currently, 25% of seniors consume cigarettes. The percentage of males who smoke ranges from 13% to 38%, whereas the percentage of females who smoke is between 1% and 16% [8]. In sum, smoking is widespread among the Saudi population, regardless of age. Similarly, a 2018 survey across 13 districts of Saudi Arabia revealed that 21.4% of the population smoked cigarettes on a regular basis [9]. Regarding the investigation of the association of smoking with vertigo, it is unclear whether there was an association between smoking and middle and inner ear disease, especially in children and adults [10,11]. Further, regarding the efficacy of the treatment for vertigo, smoking was found to reduce the efficacy of its treatment in comparison with non-smokers [12]. According to studies, vertigo is frequently associated with factors such as the female gender [13,14] and psychiatric problems such as depression [15,16] and anxiety [17]. According to the findings of extensive surveys, vertigo has a substantial impact on the quality of life and productivity at work. Nearly 50% of vertigo sufferers state that their symptoms force them to work less, and up to 12% report that their symptoms prevent them from working entirely [18]. Additionally, those who experience vertigo are more likely to fall and sustain injuries from such falls than those who do not [19].

The article "Measuring the Effect of Smoking or Tobacco Use on Vertigo Among the Adult Population in the Kingdom of Saudi Arabia" was retracted in 2023. Reasons: errors in the methods; unreliable results or conclusions; concerns about the results or conclusions.

However, given the significant effect of smoking on vertigo, which has public health implications for the population, and according to our knowledge, there are only limited data on the potential risk factors for vertigo; it is valid to conduct an extensive epidemiological investigation of the relationship between adult smoking and vertigo and the potential role of covariates (sociodemographic and chronic diseases) as determinants of the risk of vertigo in the Kingdom of Saudi Arabia.

## Materials and methods

We conducted a cross-sectional web-based survey from March 2022 to January 2023 to assess the effect of smoking on vertigo among the adult population in the Kingdom of Saudi Arabia.

The Raosoft Sample Size Calculator (Raosoft, Inc., Seattle, WA) was employed to calculate the sample size, with an expected response of 50%, a margin of error of 5%, a standard deviation of 1.96, and a total population of 25,777,851 for people aged 18-60 years, according to the General Authority for Statistics’ annual statistic for the mid-2020s in the Kingdom of Saudi Arabia. The minimum required sample size is 664. We doubled the sample size to 1,328 and added a 65% increase to decrease bias. Individuals between the ages of 18 and 60 years are considered to be within the inclusion age range, while those under 18 and those over 60 years are considered to be outside the eligibility range. After the participants were eliminated (based on the exclusion criteria), a representative sample at the national level was created from the respondents (n = 2,209).

The article "Measuring the Effect of Smoking or Tobacco Use on Vertigo Among the Adult Population in the Kingdom of Saudi Arabia" was retracted in 2023. Reasons: errors in the methods; unreliable results or conclusions; concerns about the results or conclusions.

The questionnaire was self-administered, took 5-10 minutes to finish, and had 12 items and three main sections. The sociodemographic information in the first section includes information on age, gender, place of residence, nationality, marital status, occupation, and educational attainment. While a smoking habit and the presence of chronic illnesses are found in the second part, questions involving vertigo are found in the last part. The study was carried out utilizing the software program Statistical Package for Social Sciences (SPSS) version 25.0 (IBM SPSS Statistics, Armonk, NY). Regarding descriptive statistics, the frequency and percentage for all the qualitative variables, including demographic data, were utilized. Chi-square tests were performed to evaluate the association of demographic characteristics with vertigo. The association between smoking and vertigo was also tested by the chi-square tests. The presence of vertigo (dependent variable) was predicted by binomial logistic regression that shows smoking habit as an independent variable, where odds ratios (OR) and 95% confidence intervals (CI) were calculated for each independent variable. Statistical methods were verified, assuming a significant level of p < 0.05. The results are presented in the form of tables and graphs.

The University of Hail Medical Research Ethics Committee issued its ethical approval (H-2022-310). The questionnaire was delivered to every respondent with their knowledge and consent, and any ethical issues were resolved prior to their participation.

## Results

For the study, we enrolled 2,209 adults in the Kingdom of Saudi Arabia who satisfied the eligibility criteria, comprising 1,061 males and 878 females ranging in age from 18 to 60 years. The majority (55.2%) of the participants belonged to the 18-30 age group. Of these study participants, 1,014 (45.9%) were smokers, and 308 (13.5%) used electronic cigarettes, while 908 were non-smokers (41.1%) (Table 1).

**Table 1:** General characteristics of the studied sample. ^1^A total of 122 (5.3%) had diabetes, 166 (7.3%) had hypertension, 140 (6.1%) had asthma, 96 (4.2%) had high cholesterol, 58 (2.5%) had kidney disease, 43 (1.9%) had cardiovascular disease, 36 (1.6%) had mental/psychological illness, and four (0.2%) had cancer.

Variables		n = 2,209	%
Age (years)	18-30 years	1,219	55.2
	31-40 years	574	26
	41-50 years	302	13.7
	51-60 years	114	5.2
Gender	Male	1,331	60.3
	Female	878	39.7
Marital status	Married	1,061	48
	Unmarried	1,148	52
Nationality	Saudi	2,058	93.2
	Non-Saudi	151	6.8
Region	Western	534	23.3
	Central	551	24.1
	Eastern	395	17.3
	Southern	453	19.8
	Northern	355	15.5
Educational level	Primary school	40	1.8
	Intermediate school	76	3.4
	High school	806	36.5
	Bachelor’s degree	1,194	54.1
	Master’s degree	93	4.2
Occupation	Governmental sector	617	27.9
	Private sector	540	24.4
	Retired	86	3.9
	Student	558	25.3
	Do not work	408	18.5
Chronic diseases	Yes^1^	634	28.7
	No	1,575	71.3
Smoking habit	Current smoker	1,014	45.9
	Ex-smoker	287	13
	Non-smoker	908	41.1
How many cigarettes per day?	More than 20	438	19.8
	Fewer than 20	500	22.6
	I use electronic cigarettes	308	13.5
How long have you been smoking?	More than five years	771	34.9
	Less than five years	390	17.7
	I recently quit	136	6.2

The survey’s findings indicate that smoking is more common among males than females, among people aged 18-30 years rather than people of other ages, and in the southern region than in other areas (Figures 1-3).

The article "Measuring the Effect of Smoking or Tobacco Use on Vertigo Among the Adult Population in the Kingdom of Saudi Arabia" was retracted in 2023. Reasons: errors in the methods; unreliable results or conclusions; concerns about the results or conclusions.

**Figure 1:** The distribution of smoking prevalence regarding gender differences.

**Figure 2:** The distribution of smoking prevalence regarding region differences.

**Figure 3:** The distribution of smoking prevalence regarding age differences.

Figure 4 shows that most of the participants did not suffer from vertigo while 30.80% of the participants suffered from vertigo.

**Figure 4:** Suffering from vertigo.

Table 2 shows the influence of social and demographic factors on the occurrence of vertigo. Most participants did not complain of vertigo; only 681 participants did complain of vertigo.

**Table 2:** Comparison of sociodemographic characteristics of respondents with vertigo and respondents without vertigo. *Significant

Variables		Respondents with vertigo	Respondents without vertigo	P value
Age (years)	18-30 years	342 (15.5)	877 (39.7)	0.016*
	31-40 years	196 (8.9)	378 (17.1)	
	41-50 years	101 (4.6)	201 (9.1)	
	51-60 years	42 (1.9)	72 (3.3)	
Gender	Male	415 (18.8)	916 (41.5)	0.660
	Female	266 (12)	612 (27.7)	
Marital status	Single	268 (12.1)	793 (35.9)	0.000*
	Married	413 (18.7)	735 (33.3)	
Nationality	Saudi	639 (28.9)	1,419 (64.2)	0.406
	Non-Saudi	42 (1.9)	109 (4.9)	
Region	Western	137 (6.2)	387 (17.5)	0.000*
	Eastern	104 (4.7)	262 (11.9)	
	Northern	84 (3.8)	261 (11.8)	
	Southern	242 (11)	197 (8.9)	
	Central	114 (5.2)	421 (98.8)	
Educational level	Primary school	16 (0.7)	24 (1.1)	0.000*
	Intermediate school	35 (1.6)	41 (1.9)	
	High school	275 (12.4)	531 (24)	
	Bachelor’s degree	331 (15)	863 (39.1)	
	Master’s degree	24 (1.1)	69 (3.1)	
Occupation	Do not work	108 (4.9)	300 (13.6)	0.000*
	Retired	42 (1.9)	44 (2)	
	Student	158 (7.2)	400 (18.1)	
	Private sector	209 (9.5)	331 (15)	
	Governmental sector	164 (7.4)	453 (20.5)	
Chronic diseases	Yes	349 (15.8)	285 (12.9)	0.000*
	No	332 (15)	1,243 (56.3)	

When comparing the ages of participants who suffered from vertigo, 15.5%, or most of the participants, were of the age group 18-30 years, 8.9% were 31-40 years, and 4.6% were 41-50 years. The lowest percentage of participants suffering from vertigo was in the age group 51 years and older, which was 1.9%. While there was a significant association between age and suffering from vertigo (p = 0.016), it was observed that most of the participants who appeared to suffer from vertigo were in the age group 18-30 years. For gender differences, there was no significant association between gender and suffering from vertigo (p = 393); as for the differences in marital status, there was a significant association between marital status and suffering from vertigo (p = 0.000), where it was observed that 12.1% of the participants were single and 18.7% were married, showing that married people suffer more from vertigo. There was no significant association between Saudi and non-Saudi participants with vertigo (p = 0.406). However, there was a significant correlation between the differences in the regions of Saudi Arabia and suffering from vertigo (p = 0.000); it was observed that the participants in the southern region had a higher rate of suffering from vertigo. Also, there was a significant association between the level of education and suffering from vertigo (p = 0.000); it was noted that most of the participants who suffered from vertigo were in the high school and bachelor’s level. In terms of the correlation between the differences in occupation and the presence of vertigo, it was found that the two groups who worked in the private and public sectors both faced vertigo. This indicates a significant association between occupation and the presence of vertigo (p = 0.000). Similarly, when comparing the participants who had chronic diseases and the participants who suffered from vertigo, it was noted that only a few people with chronic diseases did not suffer from vertigo, showing that there was a significant association between the presence of chronic diseases and the occurrence of vertigo (p = 0.000).

The article "Measuring the Effect of Smoking or Tobacco Use on Vertigo Among the Adult Population in the Kingdom of Saudi Arabia" was retracted in 2023. Reasons: errors in the methods; unreliable results or conclusions; concerns about the results or conclusions.

Table 3 shows the association between smoking and its factors, specifically as a risk factor for vertigo. In light of this, we found a significant association between smoking and suffering from vertigo (p = 0.000); it was noted that smokers suffered more from vertigo than non-smokers. In addition, smokers who smoked more than 20 cigarettes per day were more likely to suffer from vertigo than those who smoked less and those who use electronic cigarettes. Similarly, smokers who had smoked cigarettes for more than five years were more likely to have vertigo than those who had started smoking recently or less than five years ago. This indicates that with an increase in the number of years of cigarette smoking, there is an increase in vertigo, and if cigarette smoking continues for a longer period of time, the vertigo increases.

**Table 3:** Comparison of the smoking habit of respondents with vertigo and respondents without vertigo. *Significant

Variables		Respondents with vertigo	Respondents without vertigo	P value
Smoking habit	Non-smoker	219 (9.9)	689 (31.2)	0.000*
	Smoker	362 (14.6)	652 (29.5)	
	Ex-smoker	100 (4.5)	187 (8.5)	
How many cigarettes per day?	More than 20	182 (8.2)	256 (11.6)	0.000*
	Fewer than 20	147 (6.7)	353 (16)	
	I use electronic cigarettes	113 (5.1)	185 (8.4)	
How long have you been smoking?	More than five years	285 (12.9)	486 (22)	0.000*
	Less than five years	117 (5.3)	273 (12.4)	
	I recently quit	58 (2.9)	78 (3.5)	

In Table 4, we use binomial logistic regression to predict smoking habit as an independent variable related to vertigo when examining the association between smoking and suffering from vertigo, where it was found that 362 (14.6%) smokers were found to suffer from vertigo. The odds ratio (OR) and 95% confidence interval for vertigo in smokers were 0.257 and 0.229-0.285 (p > 0.05), which were significant predictors of vertigo.

**Table 4:** The effect of any tobacco use on the development of vertigo. Dependent variable: suffering from vertigo; predictors: (constant) smoker status OR, odds ratio; CI, confidence interval

Predictor	Total (n = 2,209)	Smoking (n = 1,014)	Non-smoking (n = 908)	OR (95% CI)	P value
Vertigo	581	362 (14.6)	219 (9.9)	0.257 (0.229-0.285)	0.000*

## Discussion

The goal of the study was to determine the prevalence of smoking habits and vertigo, as well as the relationships between them. According to the findings of our study, 1,014 out of the 2,209 individuals, or 45.9% of the sample population, were smokers. Moreover, 13% were ex-smokers. Our results show a higher prevalence of smoking in Saudi Arabia, in comparison to the recent survey that shows a lower smoking prevalence, which is equal to 12.1% [20]. Moreover, another previous study in Saudi Arabia showed that the prevalence of cigarette smoking was 21.4% in the study sample [9]. In addition to smoking’s high prevalence in the Kingdom of Saudi Arabia, demographic characteristics also contributed to variations in smoking prevalence; that is, smoking was more prevalent in the southern region than in other regions, among people between the ages of 18 and 30 years old compared to people of other ages, and among males rather than females. This was consistent with the findings of a study in which it was shown that smoking rates among adults were from 11.6% to 52.3%. The percentage of males who smoke varies from 13% to 38%, whereas the percentage of females who smoke is between 1% and 16% [8].

The article "Measuring the Effect of Smoking or Tobacco Use on Vertigo Among the Adult Population in the Kingdom of Saudi Arabia" was retracted in 2023. Reasons: errors in the methods; unreliable results or conclusions; concerns about the results or conclusions.

Furthermore, the results of another study that was done in 2018 to measure the smoking prevalence in the Kingdom of Saudi Arabia showed that the smoking prevalence among males was at 32.5% and among females at 3.9%. However, there was inconsistency and disparity in the prevalence of cigarette smoking from one region to another, in which the previous study indicated that the highest prevalence rates were found in the Al-Jawf, Northern, Riyadh, and Sharqia regions while the Asir, Jizan, and Al-Bahah regions had the lowest cigarette smoking rates [9]. As for the prevalence of vertigo, previous studies that focused on the epidemiology of vertigo and dizziness showed that their lifetime prevalence ranged from 20% to 30% [21,22]. In a previous cross-sectional study, it was found that 40.3% of the participants had at least one episode of vertigo or dizziness throughout their lifetime [23]. According to the findings of our investigation, the prevalence of vertigo was 30.80%. Comparing the demographic characteristics, we found that males more frequently experience vertigo than females and that people between the ages of 18 and 30, married people and residents of the southern region, people enrolled in high school, and people who work in the private sector more frequently experience it than others. Moreover, we found a significant association between the presence of chronic diseases and the occurrence of vertigo; a similar result was found in another study [24]. Contradicting these results, a previous study showed that females are 4.4 times more likely to suffer from vertigo [23].

Similarly, many previous studies contradict our results [16,22,25-28]. Because smoking is considered a risk factor for vertigo [29], the association of smoking with vertigo has been investigated. There was a statistically significant association between smoking and vertigo. Almost one-third of smokers suffered from vertigo. Most smokers suffering from vertigo were young; however, more than 30% of vertigo occurred in old age [14]. Also, male smokers were suffering more from vertigo than females; however, most vertigo researchers found that females are usually more affected than males [14-30]. This is an interesting finding; due to our limitations, we need more studies to focus on this difference and explain the cause of it. We found that married smokers suffered more from vertigo than single smokers, and also, smokers at the high school and bachelor’s level of education suffered more than smokers at another educational level. Smokers suffered more from vertigo than non-smokers. We found a direct relationship between the period of smoking, the number of cigarettes smoked per day, and the occurrence of vertigo. This means that with an increase in the number of cigarettes smoked and if cigarette smoking continues for a longer period, there is a higher risk of the occurrence of vertigo.

The article "Measuring the Effect of Smoking or Tobacco Use on Vertigo Among the Adult Population in the Kingdom of Saudi Arabia" was retracted in 2023. Reasons: errors in the methods; unreliable results or conclusions; concerns about the results or conclusions.

Strength and limitation

After an extensive review of the literature, to the best of our knowledge, this is the first study to measure the association between vertigo and smoking in the Kingdom of Saudi Arabia. Our study’s limitations are that it was a cross-sectional study and we used a questionnaire to collect data, so the information was subject to recall error and inaccuracy. Also, we focused on specific age groups, so pediatric and geriatric age groups were excluded. Further experimental, prospective studies with larger sample sizes in a multicenter setting would further clarify the relationship between smoking and vertigo.

## Conclusions

According to the study’s findings, adult smokers experience vertigo more than non-smokers. Additionally, demographic characteristics have been demonstrated to have a major impact on vertigo, necessitating a discussion of these issues. We anticipate that this study will highlight the need for additional research in the areas of smoking prevention and treatment, as well as the demographic characteristics and their impact on vertigo. Moreover, we need to have health promotion and smoking cessation programs and awareness about the risk of smoking.
